# Correlation between Blood Oxygen Level-Dependent Magnetic Resonance Imaging Images and Prognosis of Patients with Multicenter Diabetic Nephropathy on account of Artificial Intelligence Segmentation Algorithm

**DOI:** 10.1155/2022/5700249

**Published:** 2022-07-11

**Authors:** Yifan Zhang, Xiaohan Wang, Zhaoyu Lin, Guojian Shao, Renban Wang, Zhoutao Xie

**Affiliations:** ^1^Department of Nephrology, Wenzhou Central Hospital, Wenzhou, 325000 Zhejiang, China; ^2^Department of Radiology, Wenzhou Central Hospital, Wenzhou, 325000 Zhejiang, China; ^3^Department of Endocrinology, Wenzhou Central Hospital, Wenzhou, 325000 Zhejiang, China

## Abstract

This study was aimed to analyze the correlation between blood oxygen level-dependent magnetic resonance imaging (BOLD-MRI) images and prognosis of patients with diabetic nephropathy (DN) based on artificial intelligence (AI) segmentation algorithm, so as to provide references for diagnosis and treatment as well as prognosis analysis of patients DN. In this study, a kernel function-based fuzzy C-means algorithm (KFCM) model was proposed, and the FCM algorithm based on neighborhood pixel information (BCFCM) and the FCM algorithm based on efficiency improvement (EnFCM) were introduced for comparison to analyze the image segmentation effects of three algorithms. The results showed that the partition coefficient (V_pc_) and partition entropy (V_pe_) of the KFCM algorithm were 0.801 and 0.602, respectively, which were better than those of the traditional FCM, BCFCM, and EnFCM algorithm. At the same time, the effects of correlation between renal cortex R2∗ (RC-R2∗), renal medulla R2∗ (RM-R2∗), renal cortex D (RC-D), renal medulla D (RM-D) and renal function on the prognosis were compared. The results showed that the correlation coefficients between RC-R2∗, RM-R2∗, RC-D, RM-D and renal function were 0.57, 0.62, 0.49, and 0.38, respectively; among them, RC-R2∗ and RM-R2∗ were negatively correlated to the estimated glomerular filtration rate (eGFR), and the difference between the groups was statistically significant (*P* <0.05). Among the factors affecting the prognosis of DN patients, the GFR, hemoglobin (Hb), RC-R2∗, RM-R2∗, and RC-D were all related to the prognosis of DN, and the difference between groups was statistically obvious (*P* <0.05). It suggested that the KFCM algorithm proposed in this study showed the relatively best segmentation effect on BOLD-MRI images for DN patients; an increase in R2∗ indicated a poor prognosis, and an increase in the RC-D value indicated a better prognosis.

## 1. Introduction

Diabetes mellitus (DM) is a serious chronic disease. In recent years, with the rapid development of China's economy, people's lifestyle and eating habits have also changed rapidly. The number of DM patients is increasing [1, 2]. According to related reports, patients with DM in China accounts for more than 26% of those in the world [3, 4]. As the main target organ of DM, the kidney has also been severely affected, and its main manifestation is the occurrence of diabetic nephropathy (DN). The pathogenesis of DN is still unclear. Some scholars believe that it may be caused by the combination of genetics, renal hemodynamics, metabolism caused by hyperglycemia, hypertension, and metabolism of vasoactive substances [5]. Data show that about 40% of DM patients may develop DN, and DN is an important cause of end-stage renal disease (ESRD), second only to various glomerulonephritis [6]. Therefore, if the renal function of patients with DN can be dynamically evaluated and the prognosis of progressive decline in the renal function can be analyzed to formulate a more reasonable diagnosis and treatment plan for DN patients, this is of great significance for improving the survival rate of DN patients and improving the prognosis of patients [7].

At present, the clinical diagnosis of DN mainly relies on kidney biopsy and laboratory tests. Among them, kidney biopsy is the gold standard for diagnosis of DN, but this examination method is a traumatic examination, it is not recognized by most patients, and it is also not conducive to doctors to assess the dynamics of DN, so it is mostly no longer promoted in clinical practice [8, 9]. The laboratory examination mainly reflects the degree of renal function damage by detecting the urine microalbumin of patients with DN. However, some scientists have found that urinary microprotein cannot fully reflect renal function damage in patients with DN [10]. With the continuous development of radiology technology, functional magnetic resonance imaging (MRI) (fMRI) has inspired DN examination in terms of non-invasive examination. It is a diagnosis and treatment technology that combines MRI and computer processing. Blood oxygenation-level dependent MRI (BOLD-MRI) is established on this basis [11]. Pathophysiological studies have shown that kidney function damage caused by DM is mainly in three aspects: perfusion level, oxygenation level, and water molecule dispersion movement; and BOLD-MRI can use deoxygenated hemoglobin (Hb) as an endogenous contrast agent, which can effectively assess the oxygenation level of the tissue. On the other hand, MRI imaging can give doctors a good understanding of the anatomical structure of the patient's kidney, which can reflect changes in kidney function [1, 12]. Therefore, BOLD-MRI has the characteristics of non-radiation, non-invasiveness, and high spatial resolution, has been widely promoted in clinical practice, especially in the diagnosis and treatment of DN, and has achieved good results [13–15].

MRI image segmentation is always a difficult problem in the field of imaging. Therefore, how to improve the recognition of MRI images is an urgent problem to be solved. Fuzzy C-means algorithm (FCM) is a kind of fuzzy clustering algorithm, which is an unsupervised algorithm; and the principle of the algorithm is to continuously update the cluster center and membership function until the best cluster center cut-off is obtained [16, 17]. The FCM algorithm can be used for image segmentation based on this principle, and the best image classification result is obtained through the best clustering center. In addition, the FCM algorithm can be used for image segmentation without human intervention, and it can also effectively deal with the blurriness of the image, showing a good effect [18].

In summary, it is very necessary for the diagnosis and treatment of DN and prognostic analysis. Although the existing diagnosis and treatment techniques are feasible, there are few studies on BOLD-MRI and the prognosis of patients. Therefore, in this study, it proposed to analyze the correlation between BOLD-MRI images and prognosis of DN patients based on the kernel fuzzy c-means (KFCM) algorithm, and introduced the FCM algorithm based on neighborhood pixel information (BCFCM) and the FCM algorithm based on efficiency improvement (EnFCM) to compare with the KFCM algorithm, so as to verify their image segmentation effects; at the same time, the effects of correlation between renal cortex R2∗ (RC-R2∗), renal medulla R2∗ (RM-R2∗), renal cortex D (RC-D), renal medulla D (RM-D) and renal function on the prognosis were compared to further explore the correlation between BOLD-MRI images and prognosis of DN patients.

## 2. Materials and Methods

### 2.1. Research Objects

In this study, from June 2018 to June 2020, patients with DM and DN who met the research conditions were selected as objects from hospital. The basic clinical data of the objects during hospitalization were collected, including: name, gender, age, height, weight, body mass index (BMI), diabetes course, comorbidities, angiotensin-converting enzyme inhibitors/angiotensin receptor blockers (ACEI/ARB) medication and diuretic history. The informed consents were signed from the patients and their families. This study had been approved by the ethics committee of the hospital. Inclusion criteria of DN patients were defined as follows: all patients should meet the diagnostic criteria of DN in the Expert Consensus on DN Prevention and Treatment in the 2014 Chinese Medical Association Diabetes Branch (CDS); all patients had the first disease and were diagnosed as DN by renal biopsy; the patients and their family members had signed the informed consents. Exclusion criteria for DN patients were given as follows: DM patients with abnormal renal function that did not meet the diagnostic criteria for DN, such as kidney disease caused by hypertension; patients with serious diseases such as heart disease and blood disease; patients with severe mental illness who cannot cooperate with the trial; patients with multiple kidney stones or a single stone ≥3 mm examined by B-ultrasound; patients with multiple kidney cysts or a single cyst >3 mm; patients with incomplete clinical data; patients with contraindications to MRI examination.

### 2.2. Image Inspection and Image Processing

3.0 T magnetic resonance was adopted for scanning, using 8-channel body dedicated phased array coil. All subjects underwent conventional MRI scan, and BOLD examination obtained the coronal image of the kidney centered on the renal hilum. Before the MRI examination, it had to remove the metal objects from the patient and let the patient lie on the MRI examination table in a supine position. The noise-reducing earplugs were worn on the patient and the patient's forearms were crossed on the chest. Then, it should place the phased array coil on the patient's abdomen and ensure that the kidney can be scanned, while keeping the centerline of the coil in the same line as the midline of the abdomen. After the parameters were adjusted, the subject's feet were scanned firstly. The scan parameters were T2JJN weighted imaging on the horizontal axis, fast gradient echo sequence, and coronal T2WI-FE sequence.

BOLD used multiple gradient echo sequence and the coronal T2WI TFE sequence. The time of repeat (TR) was 100 ms, the time of echo (TE) was 3.8 ms, the field of view (FOV) was 300 × 300 mm^2^, the layer thickness was 3 mm, the slice pitch was 3.6 mm, the flip angle was 45, the bandwidth was 31.25 Hz/pixel, and the matrix was 96 × 96.

After scanning, the BOLD image was entered into the workstation. There would be two windows, one window loaded the calculated T2∗ map image, and the other window loaded the original image with a TE of 8.66 ms. Choosing an image with a smaller TE can not only ensure a clear difference in skin and medulla, but also a good signal noise ratio (SNR). Then, it had to synchronize the two windows, draw the region of interest (ROI) on the original image, and stay away from the edge area when selecting the cortical ROI to avoid the ROI from being affected by the liver, intestine, and abdominal adipose tissue at the border of the kidney. When the medullary ROI was selected, it should try to select a darker area located in the center of the renal cone. 9 ROIs were selected on the upper, middle, and lower poles of the skin and medulla of the unilateral kidney. The average value of 9 ROIs was taken as the T2∗ value of the unilateral renal cortex and medulla. According to R2∗ =1/T2∗, the RC-R2∗ value and RM-R2∗ value were calculated, and the MCR value for evaluating the oxygenation status of the entire kidney was calculated according to MCR = RM-R2∗/RC-R2∗.

### 2.3. Establishment of KFCM

FCM algorithm is widely used in image segmentation due to its unsupervised, fuzzy, and simple implementation advantages. The principle of FCM for image segmentation is as follows. If the pixel data set of the image is set as *P=*{*p*_1_, *p*_2_,...,…,*p_n_*}, where *p_i_* represents the gray value of the pixel, and *n* is the number of pixels, then the image segmentation can be simply regarded as a cluster that divides n pixels into C categories, and the cluster center of each category can be expressed as *Y=*{*y*_1_, *y*_2_,..., *y_c_*}. The basic principle of the FCM algorithm is to minimize the objective function, thereby transforming the image segmentation into the optimization of the feature function, so that the fuzzy division of n pixels can be realized. Then the objective function of the FCM algorithm can be expressed as follows:

(1) $$\begin{array}{c} K_{FCM}\left(X,Y\right)=\underset{k=1}{\overset{\text{c}}{\Sigma }}\underset{i=1}{\overset{n}{\Sigma }}u_{ik}^{s}h_{ki}^{2} \end{array}$$

(2) $$\begin{array}{c} h_{ik}={\left\|p_{i}-y_{k}\right\|}^{2} \end{array}$$

In the above equation, *s* represented the blur factor, and the size of the blur factor not only determined the blurring of the clustering, but also controlled the blur degree of the pixels between different categories. The value of *s* could not be too large or too small. If the value is too large, the fuzziness of the cluster will increase. If the value is too small, the fuzziness of clustering will reduce the result of image segmentation, which tends to be hard partitioned.

If the value of *s* is 2, the Euclidean spatial distance from pixel pi to cluster center 2 is expressed by *h_ik_*:

(3) $$\begin{array}{c} X=\left\{x_{ik},0<i<n,0<k<c\right\} \end{array}$$

In the equation (3) above, *x_ik_* represented the membership value of the pixel xi belonging to the k-th cluster center, then below equation could be obtained:

(4) $$\begin{array}{c} \underset{\left.k=1\right|}{\overset{\text{c}}{\Sigma }}x_{ik}=1,x_{ik}\in \left(0,1\right),1\leq i\leq n,1\leq k\leq c \end{array}$$

When the Lagrange multiplier method was adopted to iteratively update the K rows of the objective function, the equation was as follows:

(5) $$\begin{array}{c} F\left(X,Y,\mu \right)=\underset{k=1}{\overset{\text{c}}{\Sigma }}\underset{i=1}{\overset{n}{\Sigma }}u_{ik}^{s}h_{ki}^{2}+\mu \left(\underset{z=1}{\overset{\text{c}}{\Sigma }}u_{ik}^{s}-1\right) \end{array}$$

In the equation (5) above, *μ* was a constant, and the two first-order partial derivatives of the F function were as follows:

(6) $$\begin{array}{c} \left\{\begin{array}{c} \frac{\sigma F}{\sigma x_{ik}}=sx_{ik}^{s-1}+\mu \\ \frac{\sigma F}{\sigma y_{k}}=-2\underset{k=1}{\overset{\text{n}}{\Sigma }}x_{ik}^{s}h_{ik} \end{array}\right. \end{array}$$

The necessary conditions can be based to obtain the extreme value by the Lagrange multiplier method F function:

(7) $$\begin{array}{c} \left\{\begin{array}{c} \frac{\sigma F}{\sigma x_{ik}}=sx_{ik}^{s-1}+\mu =0\\ \frac{\sigma F}{\sigma y_{k}}=-2\underset{k=1}{\overset{\text{n}}{\Sigma }}x_{ik}^{s}h_{ik}=0 \end{array}\right. \end{array}$$

The membership degree matrix and the iterative formula of the class center thus obtained were given as follows:

(8) $$\begin{array}{c} x_{ik}={\left[\underset{z=1}{\overset{\text{c}}{\Sigma }}{\left(\frac{h_{ik}\left(p_{i},y_{i}\right)}{h_{iz}\left(p_{i},y_{k}\right)}\right)}^{2/s-1}\right]}^{-1} \end{array}$$

(9) $$\begin{array}{c} y_{k}=\frac{\underset{i=1}{\overset{\text{n}}{\Sigma }}x_{ik}^{s}p_{i}}{\underset{i=1}{\overset{\text{n}}{\Sigma }}x_{ik}^{s}} \end{array}$$

The algorithm flow after using the kernel function to improve was shown in Figure 1:

### 2.4. Observation Indicators

Laboratory indicators to be observed included serum creatinine (Scr), blood urea nitrogen (BUN), urine albumin-to-creatinine ratio (ACR), 24-hour urine albumin, 24-hour urine total protein, glycosylated hemoglobin (GHb), Hb, serum albumin, cystatin C, and superoxide dismutase.

Renal function indicators included estimated glomerular filtration rate (GFR) (eGFR), renal dynamic imaging (ECT-GFR), using EPI-GFR equation.

(10) $$\begin{array}{c} eGFR=141\times \min\left(Scr/c,1\right)\gamma \times \max{\left(Scr/c,1\right)}^{-1.209}\times 0.993^{Age}\left(\times 1.018female\right)\left(\times 1.159Black\;race\right) \end{array}$$

In the above equation, *c*: 0.7 for women and 0.9 for men; *γ*: -0.329 for women and -0.411 for men.

Image segmentation effect can be evaluated as follows. There were two image segmentation evaluation parameters used in this study, namely the Bezdek partition coefficient (V_pc_) and the partition entropy (V_pe_) [19]. The larger the value of Vpc of a clustering algorithm, the better the effect of this clustering algorithm. The equation was as follows:

(11) $$\begin{array}{c} V_{pc}=\frac{1}{n}\underset{k=1}{\overset{\text{c}}{\Sigma }}\underset{i=1}{\overset{n}{\Sigma }}x_{ki}^{2} \end{array}$$

(12) $$\begin{array}{c} V_{pc}=\frac{-1}{n}\underset{k=1}{\overset{\text{c}}{\Sigma }}\underset{i=1}{\overset{n}{\Sigma }}\left(x_{ik}\log_{2}x_{ik}\right) \end{array}$$

### 2.5. Statistical Analysis

The SPSS2.0 software was adopted for data statistical analysis, and the experimental data were expressed in terms of mean ± standard deviation (^−^x ± s). After each measurement data was tested for normality and homogeneity of variance, if the variance was uniform, the comparison between the two samples was realized by t test, the comparison of categorical data was realized by the *χ*^2^ test, and the I2 would be used to evaluate the degree of heterogeneity. *P* <0.05 indicated that there was significant difference in the data between the groups, otherwise there was no difference without statistical significance.

## 3. Results

### 3.1. General Clinical Data

57 eligible DN patients were selected in this study, including 34 males and 23 females, with an average age of 57.3 ± 6.4 years old. At the same time, 64 eligible DM patients were screened out, including 38 males and 26 females, with an average age of 56.73 ± 7.03 years old. The basic clinical data statistics were shown in Figure 2 below. Among them, the gender, age, height, and body mass index (BMI) of DN and DM patients were not significantly different (*P* >0.05). In terms of medication, no one in the DM patient group took diuretics, and about 24.8% in the DN group took diuretics; about 19.4% of DM patients took angiotensin-converting enzyme inhibitors/angiotensin receptor blockers (ACEI/ARB), and about 52.43% of DM patients took ACEI/ARB, so the difference between the two was statistically significant (*P* <0.05).

### 3.2. Statistics of Biochemical Indicators

As shown in Figure 3, the GHb of the two groups of patients were 8.21% for DN and 7.86% for DM, and there was no statistically significant difference between the two (*P* >0.05). The Hb, Cr, BUN, and eGFR of the DN group were 108.65 g/L, 186.3 *μ*ml/L, 9.7 mmol/L, and 54.65 mL/min/1.73 m^2^, respectively; while those in the DM group were 119.8 g/L, 80.04 *μ*ml/L, 3.2 mmol/L, and 92.03 mL/min/1.73 m^2^, respectively. Therefore, there were significant differences in Hb, Cr, BUN, and eGFR between the two groups of patients, showing statistical significance (*P* <0.05).

### 3.3. Comparison on the Segmentation Effects of Three Optimized Algorithms

The BCFCM algorithm [20] and EnFCM algorithm [21] were introduced for comparison. The results were shown in Figure 4. It illustrated that the Vpc values of KFCM, EnFCM, and BCFCM were all larger than those of the FCM algorithm, and the Vpe was smaller than that of the traditional FCM algorithm, and the clustering effect of the KFCM algorithm was relatively better.

### 3.4. Imaging Data of Patients

Figure 5 was the imaging data of a 45-year-old male patient with left kidney disease.  Figure 5(a) was a BOLD-MRI scan of the patient, and Figure 5(b) was an image segmented by the KFCM algorithm. Comparison of two figures revealed that the imaging effect of the BOLD-MRI image was clearer after the algorithm was optimized, which was more conducive to the diagnosis and analysis of the disease.

### 3.5. Results of RC-R2∗, RM-R2∗, and MCR Values

In this study, the RC-R2∗, RM-R2∗, and MCR of the left and right kidneys of the two groups of patients were compared, and the results were shown in Figure 6. The RC-R2∗ and RM-R2∗ of the left and right kidneys of the two groups of patients were not significantly different (*P* >0.05). The average MRC value of the DN group was 1.19, while that in the DM group was 1.35, and the difference between the two was statistically obvious (*P* <0.05).

### 3.6. Correlation Analysis between BOLD-MRI and Renal Function

In this study, the Pearson was adopted to analyze the correlation between RC-R2∗, RM-R2∗, RC-D, RM-D and the renal function (eGFR value) of patients in the DN group. The results were shown in Figure 7. The absolute value of the r coefficient of RC-R2∗, RM-R2∗, RC-D, and RM-D were 0.57, 0.62, 0.49, and 0.38, respectively. Among them, RC-R2∗ and RM-R2∗ were negatively correlated with eGFR, RC-D and RM-D were positively correlated with eGFR.

### 3.7. Multivariate Regression Analysis

The prognosis of DN patients was affected by many factors. In this study, multivariate regression analysis was performed to explore the relevant factors affecting the prognosis of patients with urinary disease and nephropathy. The clinical outcome was undertaken as the dependent variable, and eGFR, Hb, RC-R2∗, RM-R2∗, RC-D, and RM-D were undertaken as the independent variables. As shown in Table 1, the regression coefficient (*β* value), Hb, RC-R2∗, RM-R2∗, RC-D, and RM-D of eGFR were 0.95, 0.96, 1.22, 1.15, 0.91, and 0.93, respectively. Except for RM-D, the eGFR regression coefficients of eGFR, Hb, RC-R2∗, RM-R2∗, and RC-D had statistically observable differences (*P* <0.05).

## 4. Discussion

In recent years, the incidence of DM has been rising and has remained high for a long time, which has become one of the main diseases threatening human life and health. DN is one of the main chronic vascular complications of DM. In the early stage of diabetes, due to the compensatory mechanism of renal self-regulation, renal microvessels dilate, which is mainly manifested by increased eGFR [19]. With the progression of the disease, continuous high blood glucose will induce abnormal glucose metabolism, and then affect a series of metabolic disorders of lipids and proteins, and generate advanced glycation end products (AGES). AGES are mainly cleared by the kidney. Due to metabolic disorders, AGES continue to increase and the number of AGES cleared by the kidney decreases, which further leads to the accumulation of AGES in the kidney and the dysfunction of glomerular cell function. In addition, AGES also bind to receptors involved in oxidative stress and inflammatory follow-up signaling, which can lead to glomerular dysfunction. These factors interact with each other and eventually lead to thickening of glomerular basement membrane, enlargement of mesangial membrane, capillary stenosis or even occlusion, decreased renal blood flow, and decreased eGFR. Long-term effects will cause irreversible effects on the kidney [20].

Long-term chronic hypoxia is an important factor in the development of irreversible DN. Initially, direct measurement of oxygen partial pressure (PO2) using oxygen sensing electrodes inserted into renal parenchyma is the gold standard for evaluating renal oxygenation. Studies have found that oxygenated hemoglobin concentration can affect MRI signal intensity, which is called BOLD effect [21]. Subsequently, the bold-MRI technology is gradually derived from this theory [22–25]. The magnetic properties of hemoglobin in different oxygenated states are also different, deoxyhemoglobin has paramagnetism, whereas oxyhemoglobin has diamagnetism. When the concentration of deoxyhemoglobin increases, the magnetic field uniformity of surrounding tissues will be affected, resulting in a small magnetic field, resulting in a reduction of transverse relaxation time T2∗ and corresponding signal weakening in T2∗ weighted images [26–28]. After calculation (R2∗ =1/T2∗), the apparent lateral relaxation rate (R2∗ value) is obtained. The obtained R2∗ value is directly proportional to the concentration of deoxyhemoglobin, that is to say, the increase of R2∗ value means that the concentration of deoxyhemoglobin increases, which means that the oxygen partial pressure of surrounding tissues decreases. Therefore, bold-MRI can be used to assess tissue oxygenation status noninvastively [29]. This study compared and analyzed the basic clinical data of patients in the DM group and the DN group. The results showed that the number of ACEI/ARB in the DM patient group was much higher than that in the DM patient group, and the difference was statistically great (*P* <0.05). This study also analyzed the differences in biochemical indicators between the two groups of patients. The results showed that there was no visible difference in GHb between the two groups of patients, while the Hb and GFR of the DN group were greatly lower than those of the DM group, and the Cr and BUN were obviously higher than those of the DM group. The differences between the two groups were statistically significant (*P* <0.05), which was similar to the results of the study by Samoilova et al. (2020) [30]. In addition, the R2∗ values (RC-R2∗ and RM-R2∗) and MRC values of patients in the DN and DM groups were compared. The results showed that the average MRC value of the DN group was much lower than that of the DM group, and the difference was statistically significant, which further proved the feasibility of BOLD-MRI for the diagnosis and treatment of DN patients, similar to the results of Wahba et al. (2018) [31]. In this study, Pearson was used to analyze the correlation between RC-R2∗, RM-R2∗, RC-D, RM-D and renal function. At the same time, multivariate regression analysis was used to explore the related factors affecting the prognosis of patients with urinary disease and nephropathy. The results showed that RC-R2∗ and RM-R2∗ were negatively correlated with eGFR, RC-D and RM-D were positively correlated with eGFR, and eGFR, Hb, RC-R2∗, RM-R2∗, and RC-D all had an impact on the prognosis of DN patients. An increase in R2∗ indicated a poor prognosis, and an increase in D value indicated a better prognosis.

Although bold-MRI technology shows excellent performance in the diagnosis of DN, people put forward new requirements for bold-MRI with the deepening of research and more and more extensive application. In recent years, computer technology and network technology continue to develop and progress, the combination of computer technology and medical imaging technology is the development trend of medical image processing field. FCM is a popular image processing algorithm recently. At present, this algorithm is widely used in the segmentation of hemorrhagic diseases and tumors [32]. However, its application in bold-MRI image optimization of DN is almost unknown. The FCM algorithm was selected to improve the segmentation effect of BOLD-MRI images in this study. Since the traditional FCM algorithm is not ideal for image segmentation, the kernel function to optimize the original FCM algorithm to form the KFCM algorithm. In addition, the BCFCM algorithm and the EnFCM algorithm were introduced for comparison. By calculating the Vpc and Vpe of the image segmentation of the four algorithms, the image segmentation effect was compared. The results showed that the image segmentation effect of KFCM algorithm was the best.

## 5. Conclusion

In this study, a BOLD-MRI image segmentation model based on the KFCM algorithm was proposed and the BCFCM and EnFCM were introduced to improve the FCM algorithm; and the image segmentation effects of KFCM algorithm, BCFCM algorithm, and EnFCM algorithm were analyzed and compared, and applied to BOLD-MRI image segmentation of DN patients. At the same time, Pearson was used to analyze the correlation between BOLD-MRI images and prognosis of DN patients. The results showed that the segmentation performance of BOLd-MRI image by KFCM algorithm was the best, and there was a strong correlation between each index of bold-MRI image and the method rise of dn. This indicated that bold-MRI based on KFCM algorithm showed good clinical application value in diagnosis and prognosis judgment. However, the sample size of this study was small, the number of patients included was limited, and the results of the study were not overall representative. In addition, the R2∗ value was affected due to the different drugs used to control blood glucose and different blood glucose control levels in patients, and the above factors needed to be taken into consideration in future research. This study further proved that the damage of DM to the renal function of patients was multi-directional and multi-angle, and it also suggested that BOLD-MRI was helpful for diagnosis, treatment, and prognostic analysis of DN patients.

## Figures and Tables

**Figure 1:** Flow chart of FCM algorithm.

**Figure 2:** Statistics of general clinical data of patients. ∗Compared with DM group, *P* <0.05.

**Figure 3:** Statistics of biochemical indicators of patients. Hb unit was g/L, GHb unit was %, Cr unit was *μ*ml/L, BUN unit was mmol/L, and eGFR unit was mL/min/1.73 m^2^. ∗Compared with DM group, *P* <0.05.

**Figure 4:** Comparison on the segmentation effects of the three optimized algorithms.

**Figure 5:** Imaging data of a 45-year-old male patient with left kidney disease. A was the original BOLD-MRI scan, and B was the image segmented by the KFCM algorithm.

**Figure 6:** Comparison on RC-R2∗ and RC-R2∗ values. A: values of DM group; B: values of DN group; C: comparison on MCR value. ∗Compared with DM group, *P* <0.05.

**Figure 7:** Correlation analysis between BOLD-MRI and renal function. ∗Compared with eGFR, *P* <0.05.

**Table 1:** Multivariate regression analysis of prognosis of DN patients and corresponding indicators.

Independent variable	Dependent variable	*β*
eGFR	With DN or not	0.95^#^
Hb		0.96^#^
RC-R2∗		1.22^#^
RM-R2∗		1.15^#^
RC-D		0.91
RM-D		0.93

#: Compared with RC-D, P <0.05.

## Data Availability

The data used to support the findings of this study are available from the corresponding author upon request.
